# Major postoperative complications and survival for colon cancer elderly patients

**DOI:** 10.1186/1471-2482-12-S1-S20

**Published:** 2012-11-15

**Authors:** Giuseppe Grosso, Antonio Biondi, Stefano Marventano, Antonio Mistretta, Giorgio Calabrese, Francesco Basile

**Affiliations:** 1 Department “G. F. Ingrassia” Section of Hygiene and Public Health, University of Catania, Via Santa Sofia 82, 95123 Catania, Italy; 2 Department of General Surgery, Section of General Surgery and Oncology, University Medical School of Catania, Via Plebiscito 628, Catania 95121, Italy; 3 Department of Biology, Piemonte Orientale University, Alessandria, Italy

## Abstract

**Background:**

Increased life expectancy has led to elevating the mean age of the patients at the time of diagnosis of colon cancer and subsequent treatment. Differences in complication rates and outcome between elderly and younger patients have been investigated.

**Methods:**

We retrospectively analysed a database containing the information of patients who underwent surgery for stage I-III colorectal cancer from January 2004 to January 2012 at our institution and compared demographic, cancer-related, and outcomes data of 235 elderly patients with 211 patients ≤65 years old.

**Results:**

Intraoperative complications did not differ between young and old patients whereas some differences have been found in postoperative and late complications: elderly patients suffered more by ileus (P = 0.024), peritonitis or septic shock (P = 0.017), pelvic abscess (P = 0.028), wound infection (P = 0.031), and incisional/port herniation (P = 0.012) compared with younger patients. Moreover, elderly patients suffered by systemic complications such as cardiovascular (4.7% *vs*. 1.4%, P = 0.049), renal (4.7% *vs*. 0.5%, P = 0.006), and respiratory (10.6% *vs*. 5.2%, P = 0.036). The multivariate analysis assessing the odds of having a complication revealed that older age (Odd Ratio [OR] 2.75, 95% Confidential Interval [CI]: 1.67-4.52) and open surgery (OR 1.63, 95% CI: 1.01-2.62) are significantly and independently associated with having a complication.

**Conclusions:**

In our series, elderly patients have presented a slight higher incidence of comorbidities that may affect the incidence rates of postoperative complications. These results have implications in increasing the hospital stay as well as a higher rate of death.

## Background

Colorectal cancer is the third most commonly diagnosed cancer (excluding skin cancer) and the second most common cause of cancer death in the US [1,2]. Increased life expectancy has led to elevating the mean age of the patients at the time of diagnosis of colon cancer and subsequent treatment [3,4]. Since surgical techniques and multimodality treatments have improved over the years, improved rates of postoperative complications after colostomy have been achieved [5-12]. Minimally invasive surgery has demonstrated better postoperative recovery also elderly subjects, but no significant improvements have been reached in survival for these patients. Indeed, postoperative survival in the geriatric population is lower in the first year equaling that of the younger population at 5 years [13]. This group of patients presents higher rate of comorbidities that may affect their postoperative course. Actually, the indication for surgery in elderly subjects is not depending on patients’ age but by the identification and correction of known preoperative risk factors that may determine a higher rate of complications or mortality.

The aim of this study was to assess whether elderly patients significantly differs in complications and outcomes compared with younger. We examined the potential different distribution of preoperative (i.e. comorbidities), operative (i.e. surgical techniques), and post operative variables to bring the proven benefits in postoperative recovery, and analyze the factors that may influence these results.

## Methods

We retrospectively analysed a database containing the information about patients who underwent surgery for stage I-III colorectal cancer from January 2004 to January 2012 at our institution. Patients which emergency surgery was needed for an accompanying complication such as cancer perforation or failure of the self-expanding stent insertion in patients with colorectal cancer obstruction, cases in which colorectal cancer had invaded an adjacent organ or required a multiorgan surgery, and cases in which curative resection could not be performed were excluded from the study. Patients with metastatic tumors were also excluded from the analysis.

Preoperative characteristics were obtained regarding age, gender, BMI, ASA score, and comorbidities. Pathological and perioperative data regarded tumor location, type of surgical technique, operative time, blood loss, sample length, proximal and distal margin length, number of retrieved lymph nodes, tumor size, pathological differentiation and clinical stage. Postoperative data included analgesic usage, peristalsis recovery time, time until flatus, off-bed, first liquid and semi-liquid intake, and duration of hospital stay. Early and late postoperative complications were also collected.

All patients enrolled in this study were managed postoperatively by the same group of surgeons. Patients were supported by infusions in the very first several hours after surgery. After confirmation of the peristalsis recovery, liquid diet was supplied. Semiliquid diet was considered suitable for patients after report of flatus. Patients were given patient-controlled anesthesia (PCA) or short-acting drugs to control pain. Prophylactic antibiotics were used during 24-72 hours after surgery and prolonged if there was any indication of infection. The catheter was removed as early as possible except for patients with tumors located in the lower region of the rectum.

One month after surgery and every three months thereafter, physical examination, laboratory markers levels were assessed. At patient visit, symptoms were recorded and wound scars examined. Either ultrasonography or CT scan of the abdomen, in addition to chest X-ray was performed every 6 months whereas total colonoscopy was performed every year.

### Statistical analysis

Patients were divided in 2 groups according to their age (young patients aged equal or less 65 years old and elderly patients older than 65 years) and differences on variables collected were obtained. Categorical data were presented as frequencies and percentage and compared by the Chi-square test. Parametric and nonparametric continuous data were presented as mean and standard deviation and evaluated by the Student's t test and Mann-Whitney U test respectively. A *P-*value of 0.05 was considered as significant. All calculations were performed by using the SPSS software package version 17.0 (SPSS Inc., Chicago, IL).

## Results

A total of 446 patients were enrolled and analyzed in this study. Of these patients operated during the study period, 211 were equal or younger than 65 years and 235 were elderly with a mean age in the two groups of 54.6±6.6 and 76.5±6.7, respectively. No significant differences were found in the majority of the demographic parameters between the two patients groups although elderly patients were more likely to be female (*P* = 0.015), with high ASA score (*P* = 0.003) and with higher rates of minor comorbidities (*P* = 0.002) (Table 1).

Pathological parameters listed in Table 2 showed no significant differences among the two groups except that elderly receiving chemotherapy were about half than younger patients (*P* <0.001).

**Table 1:** Demographic data.

	≤65 (n=211) n (%)	>65 (n=235) n (%)	*P*
Gender			0.015
Male	115 (54.5)	101 (43)	
Female	96 (45.5)	134 (57)	
BMI			0.027
Under/normal weight	115 (54.5)	155 (66)	
Overweight	69 (32.7)	63 (26.8)	
Obese	27 (12.8)	17 (7.2)	
ASA score			0.003
1	97 (46)	69 (29.4)	
2	58 (27.5)	93 (39.6)	
3	52 (24.6)	67 (28.5)	
4	4 (1.9)	6 (2.6)	
Preoperative comorbid diseases			
Cardiovascular	77 (36.5)	114 (48.5)	0.065
Respiratory	12 (5.7)	24 (10.2)	0.080
Hepatic cirrhosis	6 (2.8)	8 (3.4)	0.735
Renal failure	8 (3.8)	18 (7.7)	0.082
Cerebral infarction	5 (2.4)	9 (3.8)	0.377
Diabetes	25 (11.8)	30 (12.8)	0.769
Autoimmunal	1 (0.5)	1 (0.4)	0.939
Others	12 (5.7)	34 (14.5)	0.002

**Table 2:** Pathological parameters.

	≤65 (n=211) n (%)	>65 (n=235) n (%)	*P*
Tumor location			0.830
Colon	129 (61.1)	146 (62.1)	
Rectum	82 (38.9)	89 (37.9)	
Tumor size (cm, mean ± SD)	4.4 ± 1.3	4.5 ± 1.5	0.595
Lymph nodes retrieved	12.2 ± 4.6	12.2 ± 4.7	0.994
Grade			0.303
Low	168 (79.6)	196 (83.4)	
High	43 (20.4)	39 (16.6)	
pT			0.121
pT1	20 (9.5)	33 (14)	
pT2	52 (24.6)	65 (27.7)	
pT3	63 (29.9)	75 (31.9)	
pT4	76 (36)	62 (26.4)	
pN			0.965
pN0	105 (49.8)	118 (50.2)	
pN1	69 (32.7)	78 (33.2)	
pN3	37 (17.5)	39 (16.6)	
TNM stage			0.915
I	39 (18.5)	47 (20)	
II	66 (31.3)	71 (30.2)	
III	106 (50.2)	117 (49.8)	
Chemotherapy	136 (64.5)	76 (32.3)	<0.001

Major differences have been found regarding intraoperative data and postoperative outcomes (Table 3). Indeed, although no differences of surgical treatment have been established between young and elderly patients, the latter had significant longer time first passing flatus (3.6 ± 2.3 *vs*. 3 ± 2.1 days, *P* = 0.004), time of first bowel motion (5.3 ± 2.4 *vs*. 4.7 ± 2.7, *P* = 0.017), time to resume normal diet (6.9 ± 2.4 *vs*. 5.1 ± 2.1, *P* <0.001), time to walk independently (5.9 ± 3.8 *vs*. 5.1 ± 3.7, *P* = 0.026), and hospital stay (12.2 ± 3.8 *vs*. 11.4 ± 2, *P* = 0.008).

**Table 3:** Intraoperative data and postoperative outcomes.

	≤65 (n=211) n (%)	>65 (n=235) n (%)	*P*
Type of operation			0.694
Laparoscopic	111 (52.6)	128 (54.5)	
Open	100 (47.4)	107 (45.5)	
Operative time (minutes)	161.8 ± 39.7	160.1 ± 36.6	0.633
Blood loss (mL)	117.8 ± 106.6	121.2 ± 109.5	0.741
Postoperative analgesic requirement (number of injections)	7.3 ±3.7	7.6 ± 3.6	0.327
Time first passing flatus (days)	3 ± 2.1	3.6 ± 2.3	0.004
Time of first bowel motion (days)	4.7 ± 2.7	5.3 ± 2.4	0.017
Time to resume normal diet (days)	5.1 ± 2.1	6.9 ± 2.4	<0.001
Time to walk independently (days)	5.1 ± 3.7	5.9 ± 3.8	0.026
Hospital stay (days)	11.4 ± 2	12.2 ± 3.8	0.008

Intraoperative complications did not differs between young and old patients whereas some differences have been found in postoperative and late complications related with surgery (Table 4). Among the major differences, elderly patients suffered more by ileus (*P* = 0.024), peritonitis or septic shock (*P* = 0.017), pelvic abscess (*P* = 0.028), wound infection (*P* = 0.031), and incisional/port herniation (*P* = 0.012) compared with younger patients. Moreover, systemic complication were even more frequent than surgery-related. Indeed, elderly patients suffering by cardiovascular, renal, and respiratory complication (4.7 to 10.6%) were at least twice than younger patients (Table 4). Furthermore, none of young patients had tromboembolism whereas the 2.1% of elderly had (*P* = 0.033). The multivariate analysis assessing the odds of having a systemic complication revealed that older age (Odd Ratio [OR] 2.75, 95% Confidential Interval [CI]: 1.67-4.52) and open surgery (OR 1.63, 95% CI: 1.01-2.62) are significantly and independently associated with having a complication (Table 5). Regarding local complications, elderly patients had 3.18 odds (95% CI: 1.71- 5.89) of having local complication compared with younger patients.

**Table 4:** Early and late complications for colorectal cancer.

	≤65 (n=211) n (%)	>65 (n=235) n (%)	*P*
Intraoperative complications			
Massive haemorrhage (>1000 ml)	1 (0.5)	1 (0.4)	0.939
Organ injury	1 (0.5)	3 (1.3)	0.369
Others	1 (0.5)	0 (0)	0.291
Post-operative complications			No
Ileus	6 (2.8)	18 (7.7)	0.024
Anastomotic haemorrhage	2 (0.9)	4 (1.7)	0.490
Abdominal haemorrhage	2 (0.9)	0 (0)	0.135
Peritonitis/septic shock	1 (0.5)	9 (3.8)	0.017
Pelvic abscess	1 (0.5)	8 (3.4)	0.028
Wound infection	3 (1.4)	12 (5.1)	0.031
Incisional/port herniation	0 (0)	7 (3)	0.012
Systemic complications			
Cardiovascular	3 (1.4)	11 (4.7)	0.049
Renal	1 (0.5)	11 (4.7)	0.006
Respiratory	11 (5.2)	25 (10.6)	0.036
Neurological	3 (1.4)	1 (0.4)	0.265
Hepatic	3 (1.4)	1 (0.4)	0.265
Urinary tract problems	5 (2.4)	16 (6.8)	0.027
Cerebral infarction	2 (0.9)	4 (1.7)	0.490
Thromboembolism	0 (0)	5 (2.1)	0.033

**Table 5:** Multivariate analysis of systemic complication.

	Systemic complications	
	
	Adjusted^a^ OR (95% CI)	*P*
Age		
≤65	1	
>65	2.75 (1.67-4.52)	<0.001
Type of operation		
Laparoscopic	1	
Open	1.63 (1.01-2.62)	0.044

^a^Adjusted for sex, BMI, TNM stage, tumor location, size and grade

As expected, the 3-year and 5-year survival rates were both higher for younger patients. Indeed, patients ≤65 years old were significantly more than patients >65 year after 3-year (82.9% *vs*. 74.5%, *P* = 0.03) and 5-year (76.3% *vs*. 67.7%, *P* = 0.043) follow-up.

## Discussion

Elderly patients represent a high percentage of patients diagnosed and treated for colon cancer due to the progressive increase in life expectancy with a consequent population aging. The results from published studies have focused on assessing differences in the outcomes obtained in such patients [13-15]. In our study we wanted to assess whether the benefits of colon surgery offers security and equal outcomes (in terms of complications) for elderly patients than those observed in younger patients, and the factors that may determine the observed differences. In the group of elderly patients we have objectified a higher percentage of local postoperative complications, mostly due to a higher number of surgical wound infections, as well as general complications, caused by urinary and respiratory infections (probably due to the removal of later catheterization and lower patient mobilization) that may influence the increase of hospital stay in the ICU admissions. Moreover, elderly patients had higher rates of cardiovascular and respiratory complications compared with younger patients. In our series, elderly patients had partially a higher incidence of associated comorbidities compared with younger, thus the higher morbidity rate in patients older than 65 years only partially maintained relationship with the prevalence of hypertension, diabetes mellitus, heart disease (significant percentage of arrhythmias and valvular disease, both degenerative diseases), and chronic bronchitis, and a worsening of the health status of older patients have been observed irrespectively of their previous conditions.

Another important finding of our study is that complications are significantly associated also with surgical technique even after adjustments with age. Several works have established the benefits of the laparoscopic approach compared with open surgery [7-11]. However, in our cohort, we observed a substantial association of complications with patients’ age even in those who underwent laparoscopid-assisted colectomy. Thus, we can not dismiss the importance of comorbidity in these patients because although still benefit from the advantages offered by the laparoscopic approach, have a higher incidence of postoperative complications than younger patients, probably largely related to the higher rate of comorbidities.

After analyzing our data, we failed in detecting potential preoperative factors that could allow us to identify a priori those patients at high risk for postoperative complications. In example, although the ASA score have been found to be higher in elderly patients (as it depends on the age and serious systemic diseases such as heart disease not incapacitating or decompensated diabetes mellitus), it was not significantly associated with higher rates of complications. Furthermore, no other preoperative factors (sex, diagnosis, staging of the lesion) or intraoperative (surgical time, blood loss, type of surgery or need for conversion to open surgery) have shown in our analysis that could consider candidates to be predictors of postoperative outcome of these patients although significant different distributions of such variables among young and old patients have been found.

## Conclusions

In our series, elderly patients have presented a slight higher incidence of comorbidity that may affect the incidence rates of postoperative complications. These results have implications in increasing the hospital stay as well as a higher rate of death. However, preoperative comorbidity rates alone can’t explain the worse outcomes in old patients. The elderly patient should be consider as a “fragile” patient and further research is needed to assess potential measure to avoid postoperative complications as well as to prolong his lifespan.

## Competing interests

The authors declare that they have no competing interests.

## Authors’ contributions

GG: conception and design, interpetration of data, writing the manuscript; AB: performed the surgery, conception and design, interpetration of data; SM: acquisition of data, data analysis, interpetration of data; AM, GC: data analysis, interpetration of data; FB: performed the surgery, given final approval of the version to be published.

## References

[B1] National Cancer InstituteCancer of the Colon and Rectumhttp://seer.cancer.gov/csr/1975_2009_pops09/index.html

[B2] American Cancer SocietyColorectal Cancer Facts and Figureshttp://www.cancer.org/acs/groups/content/@nho/documents/document/f861708finalforwebpdf.pdf

[B3] LemmensVEJanssen-HeijnenMLHoutermanSVerheijKDMartijnHPoll-FranseLCoeberghJWWhich comorbid conditions predict complications after surgery for colorectal cancer?World J Surg20073119219910.1007/s00268-005-0711-817180570

[B4] WattersJMSurgery in the elderlyCan J Surg20024510410811939651PMC3686930

[B5] BiondiAGrossoGMistrettaAMarventanoSToscanoCGruttadauriaSBasileFLaparoscopic-Assisted Versus Open Surgery for Colorectal Cancer: Short- and Long-Term Outcomes ComparisonSurgical Laparoscopy, Endoscopy & Percutaneous Techniques in press 10.1089/lap.2012.0276PMC369868623004676

[B6] BiondiATropeaABasileFClinical rescue evaluation in laparoscopic surgery for hepatic metastases by colorectal cancerSurg Laparosc Endosc Percutan Tech201020697210.1097/SLE.0b013e3181d83f0220393330

[B7] SunJJiangTQiuZCenGCaoJHuangKPuYLiangHHuangRChenSShort-term and medium-term clinical outcomes of laparoscopic-assisted and open surgery for colorectal cancer: a single center retrospective case-control studyBMC Gastroenterol2011118510.1186/1471-230X-11-8521794159PMC3160957

[B8] The Clinical Outcomes of Surgical Therapy Study GroupA comparison of laparoscopically assisted and open colectomy for colon cancerN Engl J Med2004350205020591514104310.1056/NEJMoa032651

[B9] JayneDGGuillouPJThorpeHQuirkePCopelandJSmithAMHeathRMBrownJMRandomized trial of laparoscopic-assisted resection of colorectal carcinoma: 3-year results of the UK MRC CLASICC Trial GroupJ Clin Oncol2007253061306810.1200/JCO.2006.09.775817634484

[B10] BuunenMVeldkampRHopWCKuhryEJeekelJHaglindEPahlmanLCuestaMAMsikaSMorinoMLacyABonjerHJSurvival after laparoscopic surgery versus open surgery for colon cancer: long-term outcome of a randomised clinical trialLancet Oncol20091044521907106110.1016/S1470-2045(08)70310-3

[B11] LeeJEJohYGYooSHJeongGYKimSHChungCSLeeDGKimSHLong-term Outcomes of Laparoscopic Surgery for Colorectal CancerJ Korean Soc Coloproctol201127647010.3393/jksc.2011.27.2.6421602964PMC3092077

[B12] RagusaMStatelloLMaugeriMMajoranaABarbagalloDSalitoLSammitoMSantonocitoMAngelicaRCavallaroAScaliaMCaltabianoRPriviteraGBiondiADiVMCappellaniAVasquezELanzafameSTendiECelesteSDiPCBasileFPurrelloMSpecific alterations of the microRNA transcriptome and global network structure in colorectal cancer after treatment with MAPK/ERK inhibitorsJ Mol Med (Berl)201210.1007/s00109-012-0918-822660396

[B13] Surgery for colorectal cancer in elderly patients: a systematic review. Colorectal Cancer Collaborative GroupLancet200035696897410.1016/S0140-6736(00)02713-611041397

[B14] BiondiATropeaAMonacoGMusumeciNBenfattoGBasileFManagement of early rectal cancer: our clinical experienceG Chir201132343621352705

[B15] BenfattoGBiondiADi StefanoGBasileGJiryisAStranoGMugaveroFCinardiNBenfattoSMLow rectal cancer treatment in frail elderly patients. A personal seriesG Chir20072820320817547786

